# Investigation on electronic structure, vibrational spectra, NBO analysis, and molecular docking studies of aflatoxins and selected emerging mycotoxins against wild-type androgen receptor

This article has been retracted.

**DOI:** 10.1016/j.heliyon.2021.e07544

**Published:** 2021-07-12

**Authors:** John A. Agwupuye, Peter A. Neji, Hitler Louis, Joseph O. Odey, Tomsmith O. Unimuke, Emmanuel A. Bisiong, Ededet A. Eno, Patrick M. Utsu, Tabe N. Ntui

**Affiliations:** a Department of Pure and Applied Chemistry, Faculty of Physical Sciences, University of Calabar, Calabar, Nigeria; b Department of Chemistry, Faculty of Sciences, Cross River University of Technology, Calabar, Nigeria; c Computational Quantum Chemistry Research Group, Faculty of Physical Sciences, University of Calabar, Calabar, Nigeria

**Keywords:** Mycotoxins, DFT, Structural, NBO, Molecular docking, Simulation

## Abstract

The geometry, frontier molecular orbitals (FMOs), vibrational, NBO analysis, and molecular docking simulations of aflatoxins (B1, B2, M1, M2, G1, G2), zearalenone (ZEA) emodin (EMO), alternariol (AOH), alternariol monoethyl ether (AMME), and tenuazonic acid (TeA) mycotoxins have been extensively theoretically studied and discussed based on quantum density functional theory calculations using Gaussian 16 software package. The theoretical computation for the geometry optimization, NBOs, and the molecular docking interaction was conducted using Density Functional Theory with B3LYP/6-31+G(d,p), NBO program, and AutoDock Vina tools respectively. Charge delocalization patterns and second-order perturbation energies of the most interacting natural bond orbitals (NBOs) of these mycotoxins have also been computed and predicted. Interestingly, among the mycotoxins investigated, aflatoxin G1 is seen to give the strongest stabilization energy while Zearalenone shows the highest tendency to accept electron(s) and emodin, an emerging mycotoxin gave the best binding pose within the androgen receptor pocket with a mean binding affinity of -7.40 kcal/mol.

## 1 Introduction

Most cereal and cereal-base food and feeds are reported to be contaminated with metabolites commonly called mycotoxins [1]. These mycotoxins constitute a potential threat to man and livestock. The fungi that contaminates food and feeds is the root cause of mycotoxicosis [2]. The occurrence and toxicity of both the traditionally known mycotoxins; aflatoxins (B1, B2, M1, M2, G1, G2), zearalenone (ZEA) and some emerging mycotoxins; emodin (EMO), alternariol (AOH), alternariol monoethyl ether (AMME), tenuazonic acid (TeA) has been extensively studied [1, 2, 3, 4, 5]. Quantum computational studies of mycotoxins provide information on the relationship between structure and properties and are employed in predicting the electronic structure characteristics of these compounds [6, 7, 8, 9, 10]. DFT has been used in recent times to study the reactivity of OH groups in emodin, complexation of potassium and ammonium cations with enniatin B [11, 12], tautomerism of tenuazonic acid [13], and in photophysical properties studies of zearalenone [14].

In this paper, a DFT study of the structural properties of the selected mycotoxins; AFB1, AFB2, AFG1, AFG2, AFMI, AFM2, AOH, AMME, EMO, TeA, and ZEA were investigated to comparatively elucidate the quantum chemical descriptors, account for charge transfer from NBO calculations and predicts the simulated IR spectroscopic profile of these compounds. The charge delocalization network of the investigated mycotoxins is extensively studied by performing the NBO analysis considering the natural atomic orbital occupancies, second-order perturbation energies population in the core, valence, and Rydberg sub-shell using density functional theory computations in Gaussian 16 software package [15].

Molecular docking is also performed using AutoDock Vina and Discovery Studio visualizer to further predict the biological activity of these mycotoxins and their interactions with the main target (wild-type androgen receptor (Wt AR). This computational tool is gaining prominence in toxicology and drug discovery and interaction studies [16, 17, 18, 19, 20, 21, 22, 23]. This work has further explained the chemistry of the investigated mycotoxins using quantum computational tools and will serve as a database for the preliminary study of these compounds from the quantum computational chemistry standpoint.

## 2 Computational details

The molecular structure optimization of the investigated compounds, energy, and spectroscopic profile was calculated using the DFT/B3LYP combined with basis sets 6-31G(d) and 6-311+G(d,p) in Gaussian 16 program package [15, 24] without any constraint on the geometry. The compounds were first pre-optimized with full relaxation on the potential energy surface at B3LYP/6-31G(d) basis set and re-optimized with full relaxation on the potential energy surface at B3LYP/6–3+G(d, p) basis set [25]. The HOMO-LUMO and other quantum chemical descriptors such as energy gap, hardness (ɳ), Ionization potential (IP), Electron affinity (EA), softness (σ) electronegativity (χ), electrophilicity index (ɷ), electronic potential (μ), and electronegativity (x) were calculated using the relation in Eqs. (1), (2), (3), (4), (5), (6), (7), and (8) respectively.

(1) Energy Gap (Δ*E*) = *E*_HOMO_ - *E*_LUMO_

(2) $$\eta \;=\;\frac{IP-EA}{2}$$

where

(3) $$\text{IP}=-E_{HOMO}$$

(4) $$\text{EA}=-E_{LUMO}$$

(5) $$\sigma =\;\frac{1}{\eta }$$

(6) $$\chi =\;\frac{\left(E_{HOMO+\;}E_{LOMO}\right)}{2}$$

(7) $$\omega =\;\frac{\mu^{2}}{2\eta }$$

where [26]

(8) $$\mu =-\text{x}\frac{\left(E_{HOMO+E_{LUMO}}\right)}{2}$$

The Simulated IR spectra were calculated at the B3LYP/6-31+G(d,p) [15]. To obtain holistic information patterning the population of the electrons in sub-atomic orbital coupled with the delocalization of charge and electron densities of the individual atoms in the molecules of concern, the molecular orbital calculations were carried out using NBO 3.1 program embedded in Gaussian 16 software.

## 3 Methodology

### 3.1 Construction of the ligands

The crystal structure of the wild-type androgen receptor (Wt AR) was used as a model to study the binding of high molecular weight mycotoxins. The androgen receptor protein (with its bond agonist; 5-α-dihydrotestosterone (DHT) which is its ion native ligand) was downloaded from RCSB protein data Bank (PDB ID: 4OEA) (https://WWW.rcsb.org/structure/40EA), [27]. The androgen protein receptor was optimized and edited using Biovia discovery studio [28] and AutoDock Tools version 1.5.6 sep_17_14 [29]. Water molecules were removed and the x,y, and z coordinates were set at -27.24, 2.07, and -4.42 respectively with the radius of 10.22 Å followed by the addition of polar hydrogen atoms to the amino acid residues. The protein was prepared in PDBQT format and imputed for the AutoGrid program. The 2D structures of the selected mycotoxins were sketched using the Avogadro software and geometrically optimized employing density functional theory method [15, 24], employing Becke, 3-parameter, Lee-Yang-parr correlation functional (B3LYP) method along with 6-31+G(d,p) basic set in Gaussian 16.

### 3.2 Molecular docking studies

Flexible ligand docking was performed after the preparation of the protein and the ligands (AFB1, AFB2, AFM1, AFM2, AFG1, AFG2, AOH, AMME, EMO, TeA, and ZEA). The docking calculations were carried out using the AutoDock Vina [29]. Structure stability is further validated by Ramachandran plot imbedded in the discovery studio visualizer [28] was All parameters were the same for each docking and more importantly, the pose with the highest binding mean affinity score and corresponding intermolecular interaction with the principal active site residues was chosen. Both the 3D and 2D results are shown using the discovery studio visualizer [28].

## 4 Result and discussion

### 4.1 E_HOMO-_E_LUMO_ energy gap and DFT base descriptors

The highest occupied molecular orbital (HOMO) and lowest unoccupied molecular orbital (LUMO) is quite important in quantum chemistry as they allow the investigation of stability and reactivity of molecules [26]. However, in a typical system, the HOMO acts as an electron donor, and the LUMO primarily acts as the electron acceptor [26, 30, 31]. The total energies of HOMO-LUMO and other descriptors of the investigated mycotoxins were calculated using the B3LYP/6-31+G(d,p) level. Results of the quantum chemical descriptors and illustration of their frontier molecular orbitals including the compounds are shown in Table 1 and Figure 1 respectively. The HOMO-LUMO energy gap (Table 1) of the eleven mycotoxins are arranged in decreasing order; ZEA>TeA>AOH>AFG1>AMME>AFM2>AFM1>AFB1>AFG2>AFB2>EMO.

**Table 1:** Quantum chemical descriptors of selected mycotoxins, calculated by B3LYP geometry optimization using 6-31+G(d,p) basis set.

Chemical structure	AFIBI	AFB2	AFG1	AFG2	AFM1
Energy (kJmol^−1^)	-2,810,335.62	-2,813,773.4	-3,008,039.77	-2,908072.61	-3,008,039.774
Dipole (D)	8.52	7.89	8.08	9.61	8.74
E_HOMO_ (eV)	-6.262	-6.209	-6.783	-6.444	-6.249
E_LUMO_ (eV)	-2.344	-2.298	-2.791	-2.53	-2.319
Band gap (eV)	3.918	3.911	3.912	3.914	3.93
Ionization energy	6.262	6.209	6.783	6.444	6.249
Electron affinity	2.344	2.298	2.791	2.53	2.391
Electronegativity	4.303	4.2535	4.787	4.487	4.284
Hardness	1.959	1.9555	1.996	1.957	1.965
Softness	0.26	0.26	0.25	0.26	0.26
Electrophilicity	5.38	5.16	7.77	6.26	5.28
Electronic potential	-2.344	-2.298	-2.791	-2.53	-2.319

Chemical structure	AFM2	AOH	AMME	EMO	TeA	ZEA
Energy (kJmol^−1^	-3011270.11	-2,404,749.50	-2,404,748.04	-2504140.74	-1758682.75	-2823125.75
Dipole (D)	8.37	7.27	-7.75	2.39	8.85	6.13
E_HOMO_ (eV)	-6.23	-5.84	-5.84	-6.362	-6.362	-6.11
E_LUMO_ (eV)	-2.291	-1.25	-1.229	3.003	-1.710	-1.35
Band gap (eV)	3.939	4.59	4.541	3.359	4.652	4.76
Ionization energy	6.23	5.84	5.77	6.362	6.432	6.016
Electron affinity	2.291	1.25	1.229	3.003	1.555	0.862
Electronegativity	4.2605	3.545	3.4995	4.6795	4.036	3.73
Hardness	1.19695	2.295	2.2705	1.6795	2.4385	2.577
Softness	0.25	0.22	0.22	0.29	0.21	0.19
Electrophilicity	5.17	1.79	1.79	7.57	2.95	0.96
Electronic potential	-2.291	-1.25	-1.25	-3.003	-1.555	0.862

Energy gap; E_HOMO-_E_LUMO._ E_HOMO:_ Orbital energy at highest occupied molecular orbital. E_LUMO_: Orbital energy at Lowest Unoccupied Molecular Orbital.

**Figure 1:** Optimized structures, HOMO, Energy gap, and LUMO of the studied mycotoxins (AFB1, AFB2, AFG1, AFG2, AFM1, AFM2, AOH, AMME, EMO, ZEA, and TEA respectively).

Zearalenone (ZEA), Tenuazonic acid (TeA), Alternariol (AOH), and alternariol monoethyl ether has the highest energy gap of 4.76 eV, 4.652 eV, 4.59 eV, and 4.541 eV respectively. The high energy gap of Zearalenone (4.76 eV) is in line with other reported values in the literature [14]. The total energy (-2,403.989.07 kJmol^-1^) and energy gap (4.59eV) of alternariol (AOH) agree with the results reported by [8]. AOH contains three hydroxyl groups connected to the benzochromene ring that has been reported to undergo deprotonation to anions under basic conditions and hence can exist in different tautomeric forms with high dipole moments [8, 32]. However, differences were observed in dipole moment, energy gap, ionization energy, electronegativity, electron affinity, hardness, electrophilicity, and electronic potential of all the mycotoxins studied (Table 1).

### 4.2 Vibrational analysis

Vibrational frequency calculations for Aflatoxins, zearalenone, and some emerging mycotoxins were computed using the optimized structures with its parameters through DFT, B3LYP method, and 6-31+G(d,p) basis set. Each compound have special normal vibrational mode ranging from least to highest; TeA = 78, AOH = 81, EMO = 84, AFG1 = 87, AMME = 90, AFB1 = 105, AFM1 = 108, AFB2 = 111, AFG2 = 114, AFM2 = 114, ZEA = 129 vibrations. TeA has the least number of vibrations and ZEA have the highest number of vibrations. This is due to the structural complexity, the number of functional groups, higher rotational energy, quantized energy, higher electron energy, and congestion at ground state optimization of these compounds [33]. Figure S1–S11of supporting information shows the IR spectra and collections of vibrational mode assignments for each molecule. The plotted spectra of IR were made possible by Gauss View program with 4cm^−1^ IR peak Half-width by at Half Height.

#### 4.2.1 C–H vibrations

The structure of the investigated mycotoxins which contain alkenes, aromatic, and heteroaromatic compounds shows the presence of C–H stretching vibrations though beyond the characteristics bands region of 3100–3000cm^−1^ for readily identification [34]. The bands observed were AFB1 at 3278-3029cm^−1^, AFB2 at 3251-3000cm^−1^, AFM1 at 3272-3018cm^−1^ AFM2 at 3252-3015cm^−1^, AFG1 at 3278-3017cm^−1^ AMME at 3337-3094cm^−1^ TeA at 3167-3000cm^−1^ and ZEA at 3216-3013cm^−1^ which are attributed to C–H stretching vibration as given by Gauss View IR result animation. The increase in observed bands region is due to the high absorption of quantized energy which causes rotational-vibrational transition [38]. The characteristics band region for C–H in-plane bending is observed at 1300-1000cm^−1^, with strong to weak intensity sharp bands [35]. Bands observed are AFB1 at 1170.19 and 1238.46cm^−1^ AFB2 at 1202.61cm^−1^ and 1208.54cm^−1^, AFG1 at 1201.56cm^−1^ and 1208.24cm^−1^ AFG2 at 1204.66 and 1210.02, AFM1 at 1238.57cm^−1^ AFM2 at 1238.57cm^−1^ AMME at 1183.35cm^−1^ EMO at 1073cm^−1^ AOH at 1070.20cm^−1^ TeA at 1142.69cm^−1^ and ZEA at 1138.94cm^−1^. Showing that the C–H in-plane vibration of the eleven compounds is within the standard band region [36]. However, AFM1 and AFM2 showed equal bands due to their equal vibration at the band region. The characteristics region for C–H out -of- plane bending is observed at 1000-750cm^−1^ [36]. With the help of displacement vector bands observed are; AFB1 at 841.45cm^−1^ AFB2 at 841.36cm^−1^ AFG1 at 917.42cm^−1^ AFG2 at 925.59cm^−1^ AFM1 at 841.36cm^−1^ AOH at 797.76–817.61cm^−1^, showing that C–H out-of-plane vibration of the eleven compounds is within the standard bands' region [36].

#### 4.2.2 C–O vibrations

C–O vibaration occur within 1320–1000cm^−1^ bands region for alcohol, carboxylic acids, esters and ether [37]. Using displacement vector, out of the eleven compounds ether vibration band region within 1300–1000cm^−1^ was observed for six compounds. [AFB1 at 1152.52cm^−1^, AFB2 at 1128.95cm^−1^, AFG2 at 1150.30cm^−1^, AFM1 at 1151.66cm^−1^, AFM2 at 1160.91cm^−1^, AMME at 1133.93cm^−1^] the six compounds exhibit ether functional-group vibrational character.

#### 4.2.3 C=O vibration

Acyl halides records band region within 1815–1785cm^−1^, therefore, AFB1 at 1798.83cm^−1^, AFB2 at 1797.76cm^−1^, AFM1 at 1799.34cm^−1^, AFM2 at 1798.76cm^−1^ and ZEA at 1808.18cm^−1^ and 1794.57cm^−1^ exhibit acyl halides functional group vibrational character. Also, amides bands region are within 1695–1630cm^−1^, therefore, EMO at 1689.66cm^−1^, TeA at 1678.57cm^−1^ exhibit amide functional group vibrational character. Studies shows that AFG1 at 1840.34 cm^−1^, AFG2 at 1855.41cm^−1^, AMME at 1840.49cm^−1^, and AOH at 1841.06cm^−1^ exhibit vibration beyond normal C=O vibrational modes, because quantized energy causes higher rotational-vibrational transition [38, 39].

#### 4.2.4 O–H vibrations

EMO observed vibration was at 3311.16cm^−1^ showing a strong and broad peak, while AOH at 3748.22–3731.15cm^−1^, TeA at 3732.74cm^−1,^ and ZEA at 3758.91–3732.74cm^−1^ shows region for a hydrogen bond to oxygen (OH) [39].

#### 4.2.5 C–N vibration

Amines vibration is observed at bands region 1250-1020cm^−1^ [40] vibration. The peak at 1095.00cm^−1^ was observed in TeA, showing that TeA has an amine character.

### 4.3 Natural bond orbital analysis (NBO) and natural population analysis (NPA)

The molecular orbital energies and occupancies of the mycotoxins are calculated using the B3LYP method and 6-31+G(d,p) basis set and results are presented in Table S4 and S5 of the supporting information. The energies and occupancies of the mycotoxins vary comparatively and account for delocalization of charge upon substitution corresponding to the difference in energy and orbital occupancies between the compounds as shown in Table S4 and S5 of the supporting information. The natural population analysis of the mycotoxins shows the accumulation of the charges on each of the atoms and the accumulation of electrons in the core, valence, and Rydberg. Sub-shells as seen in Table S6. The NBO analysis of the investigated mycotoxins is carried out to predict the delocalization patterns of electron density from the principal occupied Lewis-type orbitals to unoccupied non-Lewis-type orbitals (from the bonding orbitals to anti-bonding orbitals) [31, 41, 42].

The natural atomic orbital occupancies of most interacting NBO's of the selected mycotoxins together with their percentage of hybrid atomic orbitals contribution are shown in Table S4. The NBO analysis of these mycotoxins provides information aiding the investigation of the intra and intermolecular bonding as well as accounting for charge transfer [31, 43, 44, 45, 46]

#### 4.3.1 Aflatoxin B1

In AFB1molecule, the most electronegative charge of -0.56870e is accumulated on C_12_ and other atoms include: O_7_ (-0.54239e), O_15_ (-0.53577e), O_23_ (-0.53577e), O_30_ (-0.52470) and O_31_ (-0.54599). The most electropositive atoms include; C_11_ and C_16_ and C_2._ The natural pollution analysis showed that 162 electrons in the AFB1 molecule are distributed on the sub-shells (Table S6). The percentage of hybrid atomic orbitals of C_16_–O_23_, C_11_–O_15_, C_8_–C_10_, C_5_,-C_6,_ and C_1_–C_2_ of AFB1, showed that they only contributed to the p-type sub-shell as reported in Table S4. The second perturbation energies corresponding to the hyperconjugation interactions of AFB1, such as; BD(2)C_16_–O_23_ → BD∗(1)C_11_–O_15_ are considerably very large [Table 2]. The aforesaid hyper conjugative interactions are responsible for the stability of AFB1 [31, 45].

**Table 2:** Molecular docking simulation results: mean binding affinities (kcal/mol) and the important interactions.

Compound	Binding affinity	Important interaction	RMSD
AFB1	-6.50	LYS 883	1.3
AFB2	-6.74	LYS 883	0.9
AFM1	-6.53	SER703,ASP 690, HIS 689	1.4
AFM2	-7.66	SER702,ALA698,SER703,GLN693	1.2
AFG1	-6.84	SER 782,	2.9
AFG2	-6.66	GLN 783, SER 782, LYS 883	2.4
AOH	-7.17	MET 780, ASN 705, MET 742, GLY 708, GLN 711, MET 745	0.5
AMME	-6.60	GLY708, MET745, MET742	1.1
EMO	-7.40	ALA699,HIS689,GLN693 SER703, GLY688, ALA687, GLU706	0.5
ZEA	-5.7	SER703,ASP690, HIS689, SER702, ASP890	2.3
TeA	-5.58	LEU 704	0.3

#### 4.3.2 Aflatoxin B2

AFB2 compound most electronegative accumulated charge is on O_31_ atom with a charge of -0.58318e. Its most electropositive atoms are C_11_ (0.55961e) and C_16_ (0.5344e). The distribution of 164 electrons on the subshell is depicted in Table S6. It should be noted that the percentage of hybrid atomic orbitals of C_1_–C_2_, C_5_–C_6_, C_8_–C_10_, C_11_–O_15,_ and C_16_–O_23_ of AFB2 contributed to the p-type sub-shell. The stabilization energies corresponding to the hyperconjugation interactions of AFB2 responsible for the stability of these mycotoxins include; BD(_1_)C_34_–H_36_ and BD(1)C_37_–H_38_ → BD∗(1)C_34_ – H_36_ [Table S3].

#### 4.3.3 Aflatoxin G1

The most electropositive atoms in the AFG1 compound is shown to be C_14_ (0.79095e) and C_9_ (0.54868e). The most electronegative charge is accumulated on C_10_ atom (-0.5741e) (as reported in Table S5 of the supporting information). 146 electrons are distributed in the sub-shell of the molecule (Table S6). The percentage of hybrid atomic orbitals of C_1_–C_2_, C_3_–C_4_, C_9_–O_13,_ and C_14_ – O_18_ contributed to only p-type sub-shells. Other hybrid orbitals are shown in Table S4 contributed to both s-type and p-type sub-shells. The hyperconjugation interactions which are responsible for the stability of AFG1 are, BD(1) C_15_–H_16_ → BD∗(2)C_25_–C_27_, BD(1)C_30_–H_31_ → BD∗(1)C_19_–H_24_ and BD(_2_)C_3_–C_4_ → BD∗(1)C_15_–H_16._

#### 4.3.4 Aflatoxin G2

The result of the natural atomic orbital occupancies of AFG2 molecule (Table S4) showed that it’s most electronegative charge accumulate on C_21_ atom (-0.72209) and the most electropositive charges of 0.79333e and 0.79020 accumulated on C_16_ and O_7_ atoms respectively. This molecule has 163 electrons distributed in the sub-shell (Table S6). The percentage of hybrid atomic orbitals of oxygen lone pair atoms O_15_, O_20_ of AFG2 showed that they contributed to only the S-type sub-shell, and C_5_–C_6,_ C_11_–O_15_, C_16_–O_20_ contributed mainly to p-type sub-shells. The interaction energies responsible for the stability of AFG2 are shown as; BD(1)C_2_–C_3_→BD∗(1)C_11_–O_15_ and BD(1)C_2_–C_3_→BD∗(1)C_34_–H_36._ This is presented in Table S3.

#### 4.3.5 Aflatoxin M1

In the case of the AFMI compound, the most electronegative charge of -0.75723e is accumulated on the O_37_ atom ant its most electropositive charge is accumulated on C_11_ (0.55499e) and C_16_ (0.55491e) atoms. 170 electrons are distributed in the sub-shells of AFM1 as shown in Table S6 [see supporting information]. In the AFM1 molecule, the most interacting natural bond orbitals were in the C_1_–C_6_, C_4_–C_5_, C_11_–O_15_ sub-shells (Table S4). The second-order perturbation energies corresponding to the hyperconjugation interactions of AFM1 are; BD(1)C_29_–O_30_→BD∗(1)C_25_–O_37_ and BD(1)C_29_–O_31_ → BD∗(1)C_16_–O_23_ as reported in Table S3.

#### 4.3.6 Aflatoxin M2

In the AFM2 compound, the most electropositive charge (0.55171e) and the most electronegative charge (-0.75713) is accumulated on C_11_ and O_33_ respectively with 172 electrons distributed in the subshells (Table S6 of supporting information). The hybrid atomic orbitals of C_1_–C_6_, C_2_–C_3_, C_11_–O_15_, C_16_–O_23_ of AFM2 showed that they contributed maximally to the p-type sub-shells as seen in Table S4 of supporting information. The second-order stabilization energies responsible for the stability of AFM2 is shown by BD(1)C_11_–O_15_ → BD∗(1)C_35_–H_40_ and BD∗(2)C_11_–O_15_ → BD∗(2)C_16_–O_23_ (Table S3 of supporting information).

#### 4.3.7 Alternariol

The alternariol (AOH) molecule has it most electronegative charge accumulated on the C_12_ atom (-0.69420) and the most electropositive charge of 0.80073e on the C_6_ atom (Table S5 of the supporting information).134 electrons are distributed in the sub-shells of the molecule (Table S6). In AOH molecule, C_1_–C_3_, C_2_–C_5_, C_6_–O_19_, C_20_–C_23_ Hybrid orbitals contributed to only P-Type sub-shells. It is found that the interaction between bonding donor(i) orbitals LP(2)O_24,_ LP(2)O_19_ and LP(2)O_4_ with the receptor(j); BD∗(2)C_20_–C_23_, BD∗(1)O_4_–C_6_ and BD∗(2)C_6_–O_19_ of AOH is characterized with the highest stabilization energy (Table S3 of supporting information).

#### 4.3.8 Alternariol monoethyl ether

Alternariol monoethyl ether is a tautomer of AOH [8]. In this molecule, the interactions between bonding donor orbitals related to bonds of O_19_ and O_24_ and antibonding acceptor orbitals related to bonds BD∗(1)O_4_–C_6_ and BD∗(2)O_20_–C_23_ were characterized with high E(2) (energy) values which is responsible for the stability of AMME (Table S3 of supporting information). It is worthy of note that the percentage of hybrid atomic orbitals of C_1_–C_11,_ C_2_–O_15_, C_4_–O_16_, C_12_–C_13_ of AMME contributed maximally to the p-type sub-shell (Table S4 of supporting information).

#### 4.3.9 Emodin

The EMO was shown to have its most electronegative charge and highest electropositive of -0.69279 e and 0.54676 e, accumulated on C_18_ and C_2_ atoms respectively. This compound has 140 electrons distributed as shown below in the sub-shell of the molecule (Table S6 of supporting information). In EMO molecule, some of the atomic orbitals (C_1_–C_11_, C_2_–O_15_, C_4_ -C_16_, C_12_–C_13_) Contributed to only p-type sub-shells. The interaction between the bonding donor (i) orbitals with the antibonding acceptor(j) orbitals responsible for the stability of AMME are shown;

LP(1)C_3_ → BD∗(2)C_4_–O_16_, 106.37 kcal/mol

LP(1)C_6_ → BD∗(2) C_4_–O_16_), 75.50 kcal/mol

LP(2) O_22_ → LP∗(1)C_14_, 77.00 kcal/mol.

#### 4.3.10 Tenauzonic acid

TeA molecule has its most electronegative charge (-0.54063 e) accumulated on N_27_ hetero-atom with C_1_ (0.35 e) as the most electropositive atom (Table S5 of supporting information). TeA molecule also has 53 electrons distributed in the sub-shell (Table S6 of supporting formation). The percentage of hybrid atomic orbitals of oxygen lone pair atom O_31_ and C_30_–O_31_, C_1_–C_3_, C_2_–C_5,_ C_13_–O_18_, C_30_–O_31_, contributed to p-type sub-shells. The most interaction energies of 41.83 kcal/mol; (BD∗(2)C_3_–C_4_ → BD∗(2)C_19_–O_20_ and 26.60 kcal/mol; (LP(2)N_27_ → BD∗(1)C_2_–H_28_) are responsible for the stability of TeA.

#### 4.3.11 Zearalenone

In ZEA, the second-order perturbation energies corresponding to the hyperconjugation interaction; BD∗(2)C_1_–C_3_ → BD∗(2)C_2_–C_5_, LP(2) O_17_ → BD∗(2) C_13_–O_18_ and LP(2)O_18_ → BD∗(1)C_13_–O_17_ are considerably large. These interactions are most responsible for the stability of ZEA (Table 2). The most electronegative charge of -0.69149 accumulated on the C_20_ atom. On the other hand, the atom C_13_ (0.83796e) is carrying the most electropositive charge [Table 5; supporting information]. Further, the natural population analysis showed that 170 electrons in the ZEA molecule are distributed on the sub-shells (Table S6 of supporting information). It should be noted that electronegative atoms have the tendency to donate electrons whereas, electropositive atoms tend to accept electrons [44, 45, 46, 47, 48, 49, 50] Hence, AFM1 molecule has the highest electronegative charge of -0.75723 e accumulated on O_37_ and have the tendency to donate electron compared to other investigated mycotoxins. However, ZEA is found to have the highest electropositive charge of 0.83796 e on the C_13_ atom (Table S5 of supporting information). More so, the interaction between the 2-centered bond (BD(1)C_3_–C_4_) (NBO number 8) and the C_15_–H_16_ antibonding (BD∗(1)C_15_–H_16_) of AFG1 amongst other mycotoxins is seen to give the strongest stabilization energy of 95456.13 kcal/mol and the most stable Compared to other investigated mycotoxins.

### 4.4 Molecular docking of mycotoxins with wild-type androgen receptor

In this study, selected mycotoxins were used to challenge the Wt AR model to validate the agonistic activity of the chosen ligands by comparing the calculated binding pose of the investigated mycotoxins with that of DHT, a well-known ligand with characteristic positive agonist response [51]. High molecular weight mycotoxins (AFB1, AFB2, AFM1, AFM2, AFG1 AFG2, AOH, AMME, TeA, ZEA, and EMO) were successfully docked into the activate pocket (10 Å) of wild-type androgen receptor (Wt AR) and results of the most important interactions which majorly depicts conventional hydrogen bonds are shown in Figure 2. The structure stability is validated by the Ramachandran plots [52, 53, 54] as shown in Figure 3. The best binding poses were selected according to their binding affinity scores and orientation within the active site. The AutoDock vina results are shown in Table 2. Among the ligands (mycotoxins) docked within the Wt AR pocket, TeA, AFB1, and AFB2 gave the least binding scores with binding affinities of -5.87 kcal/mol, -6.50 kcal/mol and -6.74 kcal/mol respectively. Figure 2 shows the 2D interaction and Fig. S4 shows the 3D interaction [supporting information]. EMO, AOH, and ZEA were shown to have the best binding pose with binding affinities of -7.40 kcal/mol, -7.17 kcal/mol, and -5.7 kcal/mol respectively (Figure 2). The binding pose of AOH with the Amino acid residue of the wild-type androgen receptor (Arg 752, GLn711 and Asn 705) reported by [55] which correspond to the binding surrounding residue of DHT (ASn 705, GLn 711, Arg 752. And Thr 877) within the Wt AR pocket [27] and agrees with the present study (Figure 2). EMO has been experimentally shown to induce contraction in rat isolated ileum tissue by releasing endogenous acetylcholine [53]. It is capable of causing an immunosuppressive reaction which is a function of the hydrogen bond in the binding pocket of the ligands [1]. ZEA result which is the third-best binding score has earlier been reported as a qualitative method for zearalenone determination [56] due to its monovalent bonds (conventional hydrogen bonds and hydrophobic interactions) (Figure 2). The effective affinity of ZEA with target protein has been demonstrated to potentially stimulate the growth of cells with estrogenic receptors in human mammary glands [2, 57]. EMO, AOH, and ZEA are capable of inducing androgenic mutation, however, only in qualitative terms.

**Figure 2:** 2D Conformations (A) and Hydrogen bond (B) Interactions of the studied Micotoxins (4OEA_AFB1, 4OEA_AFB2, 4OEA_AFG1, 4OEA_AFG2, 4OEA_AFM1, 4OEA_AFM2, 4OEA_AOH, 4OEA_AMME, 4OEA_EMO, 4OEA_ZEA, 4OEA_TEA).

**Figure 3:** Ramachandran plots for molecular docking of the studied mycotoxins with the wild-type androgen receptor (The green dots denotes residues in the respective domains in the most favourable region which depicts the important interactions) a-k corresponds to AFB1, AFB2, AFG1, AFG2, AFM1, AFM2, AOH, AMME, EMO, ZEA, and TEA respectively.

## 5 Conclusion

In this study, the quantum chemical descriptors (HOMO-LUMO energy gap, dipole moment, total energy, etc) and vibrational analysis of selected mycotoxins were studied at DFT-B3LYP level of theory using a 6-31+G(d,p) basis set. ZEA, TeA, AOH, and AMME has the highest energy gap with ZEA having the highest number of vibrations. The NBO analysis explained the intramolecular charge transfer between the bonding and antibonding orbitals and accounts for the natural charge accumulation in the investigated mycotoxins with AFG1 having the strongest stabilization energy. The molecular docking simulation results obtained show EMO, AOH, and ZEA had the highest binding affinities within the wild-type androgen receptor pocket.

## Declarations

### Author contribution statement

John A. Agwupuye: Conceived and designed the experiments; Wrote the paper.

Peter Neji: Contributed reagents, materials, analysis tools or data.

Hitler Louis, Joseph O. Odey: Performed the experiments.

Emmanuel A. Bisiong, Ededet A. Eno, Patrick M. Utsu, Tabe N. Ntui: Contributed reagents, materials, analysis tools or data; Wrote the paper.

Tomsmith O. Unimuke: Analyzed and interpreted the data; Wrote the paper.

### Funding statement

This research did not receive any specific grant from funding agencies in the public, commercial, or not-for-profit sectors.

### Data availability statement

Data included in article/supplementary material/referenced in article.

### Declaration of interests statement

The authors declare no conflict of interest.

### Additional information

No additional information is available for this paper.

## Appendix A Supplementary data

SUPPORTING INFORMATION_V2 SUPPORTING INFORMATION_V2
